# Effect of Acupuncture on Postoperative Pain in Patients after Laparoscopic Cholecystectomy: A Randomized Clinical Trial

**DOI:** 10.1155/2023/3697223

**Published:** 2023-01-13

**Authors:** Fengxiao Wang, Pinwei Peng, Yixin Zheng, Shuqun Cheng, Yunfei Chen

**Affiliations:** ^1^Department of Acupuncture and Moxibustion, Yueyang Hospital of Integrated Traditional Chinese and Western Medicine, Shanghai University of Traditional Chinese Medicine, Shanghai, China; ^2^Department of Hepatobiliary Surgery, Yueyang Hospital of Integrated Traditional Chinese and Western Medicine, Shanghai University of Traditional Chinese Medicine, Shanghai, China

## Abstract

**Objective:**

To evaluate the efficacy and safety of acupuncture compared to that of parecoxib sodium on postoperative pain (POP), postoperative nausea and vomiting (PONV), and the Bruggemann Comfort Scale (BCS) in patients following laparoscopic cholecystectomy (LC).

**Methods:**

Eligible patients admitted to the hospital for LC were randomly allocated to either acupuncture or control groups in a 1 : 1 ratio. The subjects in the acupuncture group received acupuncture while those in the control group were injected by parecoxib sodium at their requests. The pain score, PONV score, and BCS were assessed at 0 h, 6 h, 9 h, and 12 h after operation. The primary outcome was the pain score. The secondary outcomes included the number of patients asking for parecoxib sodium from the two groups at 0–6 h and 6–12 h, PONV score, and BCS score.

**Results:**

The pain score of the acupuncture group were lower in acupuncture than that in the control group at 6 h and 9 h after operation (*P*=0.002, *P*=0.008). However, no difference was found at 12 h. Besides, the number of patients administered parecoxib sodium in acupuncture group was less than that in the control group both at 0–6 h and 6–12 h after operation (*P*=0.019, *P* < 0.001). Similarly, there were significantly lower levels of PONV score and higher levels of BCS at 6 h after operation in the acupuncture group than in the control group. However, no difference was found at 9 h and 12 h.

**Conclusion:**

Acupuncture can clinically improve the short-term treatment of postoperative pain after LC and reduce the request for extra analgesics; therefore, acupuncture might be a potential method as one of multimodal analgesia techniques to treat POP following LC. *Trial Registrations*. This trial is registered with ChiCTR2000036885 (Chinese Clinical Trial Registry).

## 1. Introduction

Laparoscopic cholecystectomy (LC), known as minimally invasive cholecystectomy [1], is currently the most favorable method for the treatment of benign gallbladder lesions such as gallbladder stones and gallbladder polyps. Compared with the open surgery, it is featured by the advantages of less trauma, fewer postoperative complications, lower mortality, shorter hospital stay, and faster recovery.

However, postoperative pain after LC remains a plague for patients, which can lead to anxiety and sleep disturbances [2], and even prolong hospitalization and recovery time [3]. So far, no unified protocol is available to provide standardized interventions for pain relief after LC. Various pharmacological and nonpharmacological measures have been clinically explored to address pain after LC, such as local anesthetics [4], transversus abdominis plane block [5], and low-pressure pneumoperitoneum [6] which needs to be further studied.

Nonsteroidal anti-inflammatory drugs (NSAIDs) are effective analgesics widely used in the postoperative surgical period. According to a systematic review, oral NSAIDs were recommended as the first line treatment for pain after LC (GRADE A), and opioids (GRADE B) were used only when necessary to avoid related side effects [7]. Notably, increasing evidence shows that NSAIDs are related to underlying risks of gastrointestinal damage and heart failure, as well as potential postsurgical complications including bleeding, anastomotic leaks, and soft tissue infection, which limits their applicable population [8].

Acupuncture is an important component of traditional Chinese medicine which has protected Chinese people against diseases for several millennia. In recent years, more and more evidence shows that acupuncture applied in the perioperative period can alleviate postoperative pain and reduce the use of opioids [9]. It had been proven effective in lots of clinical trials including total knee replacement [10], low back surgery [11], and thoracoscopic surgery [12], as a complementary and alternative therapy in conjunction with analgesic medications. Research on its mechanism shows that acupuncture can both inhibit pain by promoting the release of endogenous opioid substances in the central nervous system and block injurious signal transmission in the spinal cord by stimulating A*β* fibers in the peripheral nervous system [13]. Therefore, acupuncture analgesia might show multimodal and multitarget characters.

Yet little evidence suggests the effect of acupuncture on controlling pain after LC, and thus we designed this trial to examine the efficacy and safety of acupuncture for relieving postoperative pain in patients after LC. Simultaneously, we also estimate the influence of acupuncture on postoperative nausea and vomiting (PONV) and the levels of comfort and sedation of patients.

## 2. Materials and Methods

### 2.1. Study Design

This trial was a randomized, controlled, assessor-blinded, and single-center clinical study performed at Hepatobiliary Surgery at Yueyang Hospital of Integrated Traditional Chinese and Western Medicine, Shanghai University of Traditional Chinese Medicine (Shanghai, China).

This study had been approved by the Institutional Review Board of the Yueyang Hospital of Integrated Traditional Chinese and Western Medicine at the Shanghai University of Traditional Chinese Medicine. The reporting and design of the trial followed the Uniform Standards for Trial Reporting and the Consolidated Standard of Reporting Trials (CONSORT) [14] and Standards for Reporting Interventions in Clinical Trials of Acupuncture (STRICTA) [15]. The trial was conducted in strict accordance with the Declaration of Helsinki.

### 2.2. Subjects

The patients admitted to the hospital for LC would be screened by 2 residents. All subjects were from Yueyang Hospital of Integrated Traditional Chinese and Western Medicine affiliated to Shanghai University of Traditional Chinese Medicine from 2020 to 2022 and would receive an elective laparoscopic cholecystectomy. Inclusion criteria were as follows: patients older than 18 and no more than 75 years old, patients with American Society of Anesthesiologists (ASA) [16] grading I-II, and patients who understood and agreed to participate in the study and signed the informed consent forms. The patients would be excluded if they had local skin infections at acupoints and had nerve injuries on upper limbs or lower limbs. Those who had used analgesics before operation, who were alcoholics and who were pregnant, and those with other severe systemic diseases and serious mental illnesses would also be excluded. Moreover, patients who had participated in or were participating in other clinical trials in the past 4 weeks would not be allowed to join this trial as well.

All eligible subjects would be randomized to one of the two groups after signing their informed consent forms.

### 2.3. Randomization and Blinding

An independent statistician generated a randomization sequence by the SPSS 26.0 software. Opaque envelopes veiling the randomized number and corresponding treatment details inside were given to the subjects before they signed the informed consent forms. The acupuncturists implemented the treatments after checking the information within the envelopes. All the outcome assessors and statisticians would be blinded to the treatment details of the subjects which only the acupuncturists and statisticians who generated the randomized number knew.

### 2.4. Interventions

The procedure of the interventions and assessments is shown in Figure 1.

#### 2.4.1. Control Group

The subjects in the control group who had undergone laparoscopic cholecystectomy would be administered parecoxib sodium (drug information: parecoxib sodium for injection, H20130158, Pfizer Inc, 40 mg/dose) in a single dose, according to the actual situation.

#### 2.4.2. Acupuncture Group

*(1) Parecoxib Sodium*. The acupuncture group would receive the injection of parecoxib sodium as the same with the control group when necessary.

*(2) Preparation before Acupuncture*. Acupuncture treatments were performed by licensed acupuncturists with at least 3 years of clinical experience. All acupuncturists had received training about the treatment regimens. The acupoints chosen in this trial are shown in Table 1 (all bilateral) and Figure 2. The acupuncture protocol was determined according to the theory of traditional Chinese medicine and the consultation with specialists in this field.

*(3) Procedure of Acupuncture*. The spines of the patients would be kept in position, and skin around the acupoints would be disinfected by using 75% alcohol. The acupuncture treatment would be given when patients returned to units within 2 hours after operation. The acupuncturists would use disposable sterile needles (0.25 × 40 mm, Andy, Guizhou, China) to insert the skin with a depth of about 10–30 mm based on the acupoints' locations. Subsequently, the acupuncturists would manipulate the needles by twirling, lifting, and thrusting to get a sense of “De qi” (the feelings of soft soreness, numbness, distension, or heaviness by the patients). The same manipulations would be repeated for 3 times every 10 min. Needles would be removed softly and carefully for preventing bleeding or subcutaneous hematoma each time.

### 2.5. Outcomes Assessments

#### 2.5.1. Primary Outcome Measures

The pain score on visual analog scale (VAS) [17]: Pain intensity after LC was assessed by using a VAS at 0 h, 6 h, 9 h, and 12 h after the operation. The VAS score ranges from 0 to 10. The higher the score, the worse the pain. 0 stands for no pain, <3 for minor pain which can be tolerated, 4–6 for moderate pain that affects sleep but still tolerable, and 7–10 for severe pain which is unbearable.

#### 2.5.2. Secondary Outcome Measures

The number of patients who asked for analgesic: In this trial, parecoxib sodium would be given to the patients at their requests, and we recorded the number of them at 0–6 h and 6–12 h after LC.

The PONV on VAS score [18]: PONV score after LC was assessed at 0 h, 6 h, 9 h, and 12 h after the operation. The PONV score ranges from 0 to 10. The higher the score the worse the PONV. 0 means no nausea and vomiting, and 10 means the most nausea and vomiting.

Bruggemann comfort scale (BCS) [19]: BCS was used to assess the comfort levels of patients with scores ranging from 0 to 4. 0 stands for continuous pain; 1 for no pain at rest but serious pain while breathing deep or coughing; 2 for no pain when lying without movement and mild pain while breathing deep or coughing; 3 for no pain even with deep breath; and 4 for no pain while coughing.

### 2.6. Safety Assessments

The incidence of adverse events (AEs): Adverse events and corresponding managements would be recorded on case record form (CRF). The relationship between the AEs and interventions would be confirmed by specialists and acupuncturists. The common AEs would include needle sticking, dizziness or syncope, bleeding, the occurrence of subcutaneous hematoma, severe pain, infection, and allergy.

### 2.7. Statistical Methods

The sample size was calculated based on the changes of pain scores. The sample size was estimated based on the change in pain score on VAS at 6 h after operation. Referring to the study results of An et al. [20], the mean score of pain intensity in the acupuncture group at 6 h after operation was 3.1, with an SD of 1.1, while in the control group was 4.6, with an SD of 1.6, we made *α* = 0.05 (two-sided) and 1-*β* = 0.80, *z*_0.05/2_ = 1.96, *z*_0.2_ = 0.84 and calculated *n* = 18, and considering an attrition of 15% in total of 42 subjects were required.

An independent statistician blinded to the allocation of the subjects analyzed all the data by SPSS 26.0. *P* < 0.05 (two-tailed) was considered statistically significant. Enumeration data were described by frequency or percentage and tested by *χ*^2^ or Mann–Whitney *U* rank sum test. Measurement data were described by means ± SD or medians (Min, Max). Student's *t*-test, multivariate analysis of variance and Mann–Whitney *U* rank sum test was used for the between-group comparisons.

### 2.8. Data Management and Quality Control

The outcome assessors were trained before the trial and would begin to record the patients' information and the results of observed indicators on the CRF after each visit. To ensure the accuracy, two researchers are separately responsible for entering the data extracted from the CRFs into Excel. The personal and hospitalization information of the subjects, including name, age, gender, ID, and telephone number, as well as surgery details would be confidential.

Experts in surgery, acupuncture, anesthesiology, statistics, and methodology were involved in the development, review, and revision of this study protocol. Specified introduction and training were given to different participants involved in the trial, such as patient recruitment, communication techniques, completion of the CRF, interventions, data management, and analysis. Any reason for discontinuation of the trial would be recorded in the CRFs.

## 3. Results

### 3.1. Demographic Characteristics

60 were eligible for the inclusion criteria, of whom 18 were excluded due to failures in further screening. 42 participants were randomly assigned to either the acupuncture group or control group with 21 for each. Finally, a total of 42 subjects were analyzed (Figure 3).

In Table 2 shows the demographic characteristics of the subjects. Showing no significant differences in age, sex, body mass index, ASA, occupation, education level, and concomitant diseases.

### 3.2. Efficacy

#### 3.2.1. Primary Outcome Assessments

Both the pain scores on VAS decreased in the two groups after their treatments (Table 3). Pain score decreased from 5.67 to 1.86 in the acupuncture group, while from 5.76 to 1.90 in the control group. At 6 h and 9 h after operation, the difference between the two groups was statistically significant (*P*=0.002, *P*=0.008). There was no difference observed at 12 h between the two groups (*P* > 0.05).

#### 3.2.2. Secondary Outcome Assessments

As to the number of patients required for parecoxib sodium, the difference between the two groups were statistically significant both in 0–6 h and 6–12 h after operation (*P*=0.019, *P* < 0.001) (Table 4).

PONV scores in the two groups decreased after their treatments (Table 3). PONV score decreased from 4.10 to 1.57 in the acupuncture group, as from 4.38 to 1.43 in the control group. At 6 h after operation, the difference between the two groups was statistically significant (*P*=0.004). However there was no difference in PONV score was found at 9 h and 12 h (*P* > 0.05).

The results of BCS are shown in Table 5. After treatments, higher BCS scores were recorded in both groups. At 6 h after operation, the difference between the two groups was statistically significant in BCS score (*P*=0.007). However, there was no difference in BCS score was found at 9 h and 12 h (*P* > 0.05).

### 3.3. Adverse Events

During the study, 3 subjects experienced bleeding after removing the needles but that lasted for less than 30 seconds with no discomfort, and 2 subjects had subcutaneous hematoma after bleeding. Besides there is no severe adverse events related to acupuncture and parecoxib sodium (Table 6).

## 4. Discussion

To our knowledge, this RCT was the first to explore the effectiveness of an acupuncture treatment regimen aimed at POP in patients after LC both subjectively and objectively. We found that acupuncture can help relieve POP, especially in a short period after LC, and reduce the number of patients required for extra analgesics. Moreover, acupuncture can also improve the comfort levels of patients and alleviate their PONV. The results of this trial supported that acupuncture might be an adjunctive method for the initial management for LC.

### 4.1. Laparoscopic Cholecystectomy and POP

With the advancement of techniques, laparoscopic cholecystectomy has gradually replaced traditional open cholecystectomy in most occasions [21] and been clinically used for almost 40 years. LC can decrease but not yet eliminate postoperative pain which remains a troublesome problem affecting patients psychologically and physiologically and causing nausea, vomiting, etc. The pains after LC are mainly classified as follows [22]: parietal pain caused by traumatic surgery and the placement of drainage tube [23], visceral pain due to the gallbladder and nearby nerves being stretched and damaged, and shoulder and back pain mainly related to diaphragmatic irritation resulting from CO_2_ pneumoperitoneum during the surgery [22]. Since the mechanisms of postoperative pain are multifactorial, a single analgesic approach might be inadequate. Consequently, a combination of two or more treatment approaches are required to alleviate postoperative pain after LC. But currently, more evidence and data are needed to support the efficacy of multimodal analgesia for LC.

### 4.2. The Analgesic Effect and Regimen of Acupuncture

Acupuncture is one of the most ancient medical treatments. Acupuncturists treat diseases by inserting needles into the meridians and acupoints on the skin with certain manipulations. The analgesic effect of acupuncture has drawn much attention, and numerous studies about it have been conducted since the 1970s. There are more than 80 recommendations related to acupuncture in about thirty-nine guidelines by the National Guideline Clearinghouse (NGC), of which 49 explicitly recommend acupuncture for medical practice and 37 (75.51%) are about the treatment of painful conditions by acupuncture [24]. What merits attention is that, in the perioperative period, acupuncture combined with anesthetics and analgesics has the following advantages [9]: (i) enhancing the analgesic effect, (ii) reducing the dosage of anesthetics and analgesics, (iii) reducing the side effects of anesthetics and analgesics such as dizziness, nausea and vomiting, intestinal distention, and urinary shutdown; (iv) protecting organs including the heart and brain; and (v) shortening the recovery time of patients after surgery.

Accordingly, we designed this study to examine the efficacy of acupuncture in treating postoperative pain compared to that of parecoxib sodium recommended by clinics for patients following LC by comparing the VAS scores of pain and the proportion of patients asked for parecoxib sodium. In addition, we also examined the effect of acupuncture on PONV and levels of comfort.

The acupuncture protocol in this trial was based on the theory of TCM and clinical experience. In the theory of acupoints, “Jing-river Points” is a generic term of Jing, Xing, Shu, Yuan, Jing, and He points of each meridian, describing meridian Qi as water flowing from small to large. GB 41 is the Shu point of the gallbladder meridian, while GB 34 is the He point. Shu point has a good effect on pain conditions, and He point is mainly used for treating diseases of Zang-fu organs. So, we chose the GB 41 and GB 34 to treat the pain following LC. TE 5 is the Luo point that connects the triple energizer meridian and gallbladder meridian, and both TE 5 and LI 4 are commonly used to manage pain and postoperative nausea and vomiting which might be related to the stimuli-specific cortical networks [25, 26].

### 4.3. Pain Score

In this study, we measured the pain intensity with a VAS. There was a significant reduction in pain score in the acupuncture group compared with the control group at 6 h after operation, although no difference was found in rescue analgesia between the two groups in 0–6 h after operation, indicating that acupuncture might have an extra analgesia effect compared with rescue analgesia. And the effect of acupuncture lasted until 9 h after operation, as the VAS of pain score was still lower in the acupuncture group than in the control group. However, there was no significant difference between the two groups in pain score at 12 h after operation. On the one hand, the request of rescue analgesia in the control group was higher compared to the acupuncture group in the 6–12 h after operation that might minimize the difference of pain score between the two groups. On the other hand, the pain score in both groups was less than 3 points which means minor pain that can be tolerated implying that the analgesia effect of acupuncture was comparable to the parecoxib sodium in the 6–12 h after operation.

Besides, the pain score decreased by 3.81 points at 12 h after operation. It has been reported that a reduction of 2 points in the VAS score reflected satisfactory pain relief in patients after surgery [27]. Our results were consistent with relevant studies. Topdemir EA and her colleagues [28] found that acupressure was effective for reducing postoperative pain and increasing comfort as well as improving gastrointestinal function after LC. Taras I. Usichenko and his colleagues [29] found that acupuncture combined with standard pain treatment produced an extra 1.6 points reduction compared to the standard care group, and they recommended acupuncture as a routine and supplemental therapy for pain management after elective cesarean delivery. In the Crespin's et al. research [30], acupuncture used in total joint replacement reduced the self-reported pain by 1.91 points and alleviated pain in a short period. Gabriel J Tsao [31] also reported that the acupuncture group in their study enjoyed greater relief in pain after tonsillectomy compared with the control group, and the difference between the postoperative pain scores of the two groups was clinically significant.

### 4.4. The Request of Parecoxib Sodium

In terms of extra analgesics, the proportion of patients required for parecoxib sodium in the acupuncture group was smaller than that in the control group at 0–6 h and 6–12 h after operation in our study. The need for additional analgesics has been reported to vary widely among individuals following LC, with approximately 10–30% of the patients requiring no additional analgesics [32]. Our study showed that acupuncture reduced the demands for additional analgesics after LC compared with the control group. Langenbac applied acupuncture for haemorrhoidopexy patients to manage postoperative pain, and the results showed that the rescue analgesics used in the acupuncture group were less than those used in the sham acupuncture and conventional groups. So, they concluded that acupuncture might be an adjunct therapy to conventional analgesia [33]. Wang et al. and his colleagues observed that transcutaneous electric acupoint stimulation decreased the consumption of remifentanil by 39% compared to the control group and reduced the anesthesia-related side effects after surgery. They suggested that, in the future, more studies would be set up to explore different acupoints for relieving postoperative pain caused by different types of operations according to the parts of the body [34].

### 4.5. PONV Score and BCS Score

PONV might be related to the trauma of surgery and anesthesia, as well as the analgesia. We found that the PONV score in the acupuncture group was lower than that in the control group at 6 h after operation. In a systematic review, acupuncture along with and after tonsillectomy can reduce the incidence of PONV in the acupuncture group compared to the control group [35]. Stoicea et al. thought that the antiemetic effect of acupuncture might be related to the release and modulation of opioid neuropeptides [36]. Ferrari and Broughton added that anxiolytics might mediate the antiemetic effect of acupuncture [37]. Nevertheless, due to the difference of demands for parecoxib sodium between the two groups mentioned above, it is hard to conclude that acupuncture can reduce PONV after LC as side effects of analgesics might cause PONV. As for the levels of comfort, our study found that acupuncture can improve the comfort level at 6 h after operation. After reviewing relevant literature, we found little research to investigate the effect of acupuncture on comfort. A similar study conducted by Unulu and Kaya found that acupressure on the Neiguan acupoint (PC 6) in the postoperative period enhanced the comfort level of the patient [38]. Fanti et al. found that acupuncture can decrease the discomfort and anxiety levels of patients as well as reduce the consumption of sedative drugs and their related adverse effects [39]. However, contrary to the above results, Chen et al. found that transcutaneous electrical acupoint stimulation (TEAS) in lung cancer surgery did not reduce Observer's Assessment of Alertness/Sedation (OAAS) score compared to the control group in their study [12].

### 4.6. Limitations

This study had some limitations. Firstly, there was an absence of a sham acupuncture group as the control group. This trial aimed to examine the efficacy and safety of acupuncture for postoperative pain by comparing it to that of parecoxib sodium, so we did not set up the sham acupuncture group. Secondly, we performed acupuncture after the patients returned to the units, resulting in a time difference for completing acupuncture treatment between patients. To deal with this problem, the acupuncturists were asked to come to the units and implement acupuncture as quickly as they received the information within 2 h after operation. Thirdly, the observation time was limited, and no follow-up investigation was involved after the discharge. Thus, the long-term analgesic effect of acupuncture and the optimal acupuncture frequencies remain unknown. Fourthly, this was a single single-center trial, and the sample size was small that might introduce potential biases. Despite this, the outcomes of this trial will be used to guide a better design including multicenter and sample size calculation for a further randomized controlled trial. Finally, all the patients in the acupuncture group received the same standard regimen of acupuncture; however, semistandard regimen which is one of the features of TCM was more widely used in clinics [40]. In the future, we will introduce a sham acupuncture group to examine the nonspecific effects of acupuncture. Moreover, we will expand the observation period to observe the long-term effect of acupuncture as well as explore the optimal acupuncture frequencies of for patients undergoing LC. Besides, a semistandard prescription of acupuncture treatment will be applied for the patients.

## 5. Conclusions

The results of this trial serve as clinical evidence supporting the fact that acupuncture is safe and provides a short-term analgesic effect for patients following LC at least in the 12 h after operation. Overall, our paper suggests that acupuncture might be a potential method as one of the multimodal analgesia techniques to deal with POP following LC.

## Figures and Tables

**Figure 1:** The procedure of interventions and assessments.

**Figure 2:** Locations of the acupoints.

**Figure 3:** Flow chart diagram.

**Table 1:** Locations of acupoints in the acupuncture group.

Acupoint	Location
Hegu (LI4)	On the dorsum of the hand, radial to the midpoint of the second metacarpal bone
Waiguan (TE 5)	On the posterior aspect of the forearm, midpoint of the interosseous space between the radius and the ulna, and 2 cun^a^ proximal to the dorsal wrist.
Yanglingquan (GB 34)	On the fibular aspect of the leg and in the depression anterior and distal to the head of the fibula
Zulinqi (GB 41)	On the dorsum of the foot, distal to the junction of the bases of the fourth and fifth metatarsal bones, and in the depression lateral to the fifth extensor digitorum longus tendon

^a^1 cun (≈20 mm) is defined as the width of the interphalangeal joint of patient's thumb.

**Table 2:** Demographic characteristics of the participants.

	Acupuncture group (*n* = 21)	Control group (*n* = 21)	*P* value
Age^a^ (y)	57.75 ± 11.64	56.60 ± 11.76	0.752
Sex^b^ (M/F)	10/11	8/13	0.533
BMI^b^, *N*	—	—	0.552
Normal weight	13	15	
Overweight	5	5	
Obesity	3	1	
ASA^b^, *N* (%)	—	—	0.694
I	16 (47.1)	18 (52.9)	
II	5 (62.5)	3 (37.5)	
Occupation^b^, *N* (%)	—	—	0.537
Employed	12 (57.1)	10 (47.6)	
Retired	9 (42.9)	11 (52.4)	
Education level^b^, *N* (%)			0.371
≤High school	5 (23.8)	8 (38.1)	
≥College degree	16 (76.2)	13 (61.9)	
Concomitant diseases^b^, *N* (%)	12 (57.1)	13 (61.9)	0.753

**Table 3:** Pain and PONV scores at 0 h, 6 h, 9 h, and 12 h.

Outcomes	Acupuncture group (*n* = 21)		Control group (*n* = 21)		*P* value^a^
	Mean (SD)	Change from 0 h mean (SD)	Mean (SD)	Change from 0 h mean (SD)	
Pain score					
0 h	5.67 (1.28)		5.76 (1.30)		0.812
6 h	4.38 (0.97)	−1.29 (0.58)	5.45 (1.08)	−0.31 (0.37)	0.002
9 h	2.05 (0.88)	−3.62 (1.90)	2.76 (0.77)	−3.00 (0.92)	0.008
12 h	1.86 (0.99)	−3.81 (1.62)	1.90 (1.17)	−3.85 (1.70)	0.887
PONV score					
0 h	4.10 (1.30)		4.38 ± 1.27		0.476
6 h	3.10 (0.87)	−1.00 (0.61)	4.00 ± 1.04	−0.38 (1.30)	0.004
9 h	3.92 (1.22)	−0.16 (1.58)	4.24 ± 1.17	−0.14 (1.58)	0.398
12 h	1.57 (0.75)	−2.52 (0.60)	1.43 ± 0.83	−2.95 (1.62)	0.560

PONV, postoperative nausea and vomiting; ^a^calculated using multivariate analysis of variance.

**Table 4:** The number of patients required for parecoxib sodium (%).

	Acupuncture group (*n* = 21)	Control group (*n* = 21)	*P* ^*a*^
0–6 h	3 (14.29)	10 (47.62)	0.019
6–12 h	2 (9.52)	6 (28.57)	<0.001

Data are presented as the number (%). ^*a*^calculated using Pearson's chi-square test.

**Table 5:** BCS scores at 0 h, 6 h, 9 h, and 12 h.

	Acupuncture group (*n* = 21)	Control group (*n* = 21)	*P* value^a^
BCS score			
0 h	1 (0, 3)	1 (0, 3)	0.884
6 h	2 (0, 4)	1 (0, 2)	0.007
9 h	2 (1, 3)	2 (0, 3)	0.396
12 h	3 (2, 4)	3 (2, 4)	0.383

Data are presented as the median (min,max). ^a^Calculated using Mann–Whitney *U* rank sum test.

**Table 6:** Adverse events related to intervention.

	Acupuncture group (*n* = 21)	Control group (*n* = 21)
Adverse event		
Overall	5	0
Severe adverse events	0	0
Bleeding	3	0
Subcutaneous hematoma	2	0
Infection and allergy	0	0

^a^adverse events were counted by type rather than frequency in the same subject.

## Data Availability

The datasets that support our findings in the study are available from the corresponding author upon reasonable request.

## References

[1] Kim S. S., Donahue T. R. (2018). Laparoscopic cholecystectomy. *JAMA*.

[2] Haack M., Simpson N., Sethna N., Kaur S., Mullington J. (2020). Sleep deficiency and chronic pain: potential underlying mechanisms and clinical implications. *Neuropsychopharmacology*.

[3] Rosero E. B., Joshi G. P. (2017). Hospital readmission after ambulatory laparoscopic cholecystectomy: incidence and predictors. *Journal of Surgical Research*.

[4] Rutherford D., Massie E. M., Worsley C., Wilson M. S. (2021). Intraperitoneal local anaesthetic instillation versus no intraperitoneal local anaesthetic instillation for laparoscopic cholecystectomy. *Cochrane Database of Systematic Reviews*.

[5] Grape S., Kirkham K. R., Akiki L., Albrecht E. (2021). Transversus abdominis plane block versus local anesthetic wound infiltration for optimal analgesia after laparoscopic cholecystectomy: a systematic review and meta-analysis with trial sequential analysis. *Journal of Clinical Anesthesia*.

[6] Ko-Iam W., Paiboonworachat S., Pongchairerks P., Junrungsee S., Sandhu T. (2016). Combination of etoricoxib and low-pressure pneumoperitoneum versus standard treatment for the management of pain after laparoscopic cholecystectomy: a randomized controlled trial. *Surgical Endoscopy*.

[7] Barazanchi A. W. H., MacFater W. S., Rahiri J. L. (2018). Evidence-based management of pain after laparoscopic cholecystectomy: a PROSPECT review update. *British Journal of Anaesthesia*.

[8] Zhao-Fleming H., Hand A., Zhang K. (2018). Effect of non-steroidalanti-inflammatory drugs on post-surgical complications against the backdrop of the opioid crisis. *Burns Trauma*.

[9] Yuan W., Wang Q. (2019). Perioperative acupuncture medicine: a novel concept instead of acupuncture anesthesia. *Chinese Medical Journal*.

[10] Chen C. C., Yang C. C., Hu C. C., Shih H. N., Chang Y. H., Hsieh P. H. (2015). Acupuncture for pain relief after total knee arthroplasty: a randomized controlled trial. *Regional Anesthesia and Pain Medicine*.

[11] Cho Y. H., Kim C. K., Heo K. H. (2015). Acupuncture for acute postoperative pain after back surgery: a systematic review and meta-analysis of randomized controlled trials. *Pain Practice*.

[12] Chen J., Zhang Y., Li X. (2020). Efficacy of transcutaneous electrical acupoint stimulation combined with general anesthesia for sedation and postoperative analgesia in minimally invasive lung cancer surgery: a randomized, double-blind, placebo-controlled trial. *Thoracic Cancer*.

[13] Coutaux A. (2017). Non-pharmacological treatments for pain relief: TENS and acupuncture. *Joint Bone Spine*.

[14] Schulz K. F., Altman D. G., Moher D., For the CONSORT Group (2010). CONSORT 2010 statement: updated guidelines for reporting parallel group randomised trials. *BMJ*.

[15] MacPherson H., Altman D. G., Hammerschlag R. (2010). Revised standards for reporting interventions in clinical trials of acupuncture (STRICTA): extending the CONSORT statement. *Journal of Alternative & Complementary Medicine*.

[16] Hackett N. J., De Oliveira G. S., Jain U. K., Kim J. Y. (2015). ASA class is a reliable independent predictor of medical complications and mortality following surgery. *International Journal of Surgery*.

[17] Reed M. D., Van Nostran W. (2014). Assessing pain intensity with the visual analog scale: a plea for uniformity. *The Journal of Clinical Pharmacology*.

[18] Kunzli B. M., Walensi M., Wilimsky J. (2019). Impact of drains on nausea and vomiting after thyroid and parathyroid surgery: a randomized controlled trial. *Langenbeck’s Archives of Surgery*.

[19] Yao Z. Y., Jia Z., Xie Y. H. (2017). Analgesic effect of dezocine in different doses on elderly patients undergoing abdominal operation under general anesthesia and its influence on stress response to postoperative tracheal extubation. *European Review for Medical and Pharmacological Sciences*.

[20] An L. X., Chen X., Ren X. J., Wu H. F. (2014). Electro-acupuncture decreases postoperative pain and improves recovery in patients undergoing a supratentorial craniotomy. *The American Journal of Chinese Medicine*.

[21] Okamoto K., Suzuki K., Takada T. (2018). Tokyo guidelines 2018: flowchart for the management of acute cholecystitis. *Journal of Hepato-Biliary-Pancreatic Sciences*.

[22] Choi G. J., Kang H., Baek C. W., Jung Y. H., Kim D. R. (2015). Effect of intraperitoneal local anesthetic on pain characteristics after laparoscopic cholecystectomy. *World Journal of Gastroenterology*.

[23] Qiu J., Li M. (2018). Nondrainage after laparoscopic cholecystectomy for acute calculous cholecystitis does not increase the postoperative morbidity. *BioMed Research International*.

[24] Guo Y., Zhao H., Wang F. (2017). Recommendations for acupuncture in clinical practice guidelines of the national guideline clearinghouse. *Chinese Journal of Integrative Medicine*.

[25] Fernandez Rojas R., Liao M., Romero J., Huang X., Ou K. L. (2019). Cortical network response to acupuncture and the effect of the hegu point: an fNIRS study. *Sensors*.

[26] Yang J., Zeng F., Feng Y. (2012). A PET-CT study on the specificity of acupoints through acupuncture treatment in migraine patients. *BMC Complementary and Alternative Medicine*.

[27] Myles P. S., Myles D. B., Galagher W. (2017). Measuring acute postoperative pain using the visual analog scale: the minimal clinically important difference and patient acceptable symptom state. *British Journal of Anaesthesia*.

[28] Topdemir E. A., Saritas S. (2021). The effect of acupressure and reiki application on patient’s pain and comfort level after laparoscopic cholecystectomy: a randomized controlled trial. *Complementary Therapies in Clinical Practice*.

[29] Usichenko T. I., Henkel B. J., Klausenitz C. (2022). Effectiveness of acupuncture for pain control after cesarean delivery: a randomized clinical trial. *JAMA Network Open*.

[30] Crespin D. J., Griffin K. H., Johnson J. R. (2015). Acupuncture provides short-term pain relief for patients in a total joint replacement program. *Pain Medicine*.

[31] Shah A. N., Moore C. B., Brigger M. T. (2020). Auricular acupuncture for adult tonsillectomy. *The Laryngoscope*.

[32] Wills V. L., Hunt D. R. (2002). Pain after laparoscopic cholecystectomy. *British Journal of Surgery*.

[33] Langenbach M. R., Aydemir-Dogruyol K., Issel R., Sauerland S. (2012). Randomized sham-controlled trial of acupuncture for postoperative pain control after stapled haemorrhoidopexy. *Colorectal Disease*.

[34] Wang H., Xie Y., Zhang Q. (2014). Transcutaneous electric acupoint stimulation reduces intra-operative remifentanil consumption and alleviates postoperative side-effects in patients undergoing sinusotomy: a prospective, randomized, placebo-controlled trial. *British Journal of Anaesthesia*.

[35] Cho H. K., Park I. J., Jeong Y. M., Lee Y. J., Hwang S. H. (2016). Can perioperative acupuncture reduce the pain and vomiting experienced after tonsillectomy? A meta-analysis. *The Laryngoscope*.

[36] Stoicea N., Gan T. J., Joseph N. (2015). Alternative therapies for the prevention of postoperative nausea and vomiting. *Frontiers of Medicine*.

[37] Ferrari L., Broughton N. (2016). Possible mechanism(s) for acupressure PONV prophylaxis. *British Journal of Anaesthesia*.

[38] Unulu M., Kaya N. (2018). The effect of Neiguan point (P6) acupressure with wristband on postoperative nausea, vomiting, and comfort level: a randomized controlled study. *Journal of Peri Anesthesia Nursing*.

[39] Fanti L., Gemma M., Passaretti S. (2003). Electroacupuncture analgesia for colonoscopy. A prospective, randomized, placebo-controlled study. *American Journal of Gastroenterology*.

[40] Lin L. L., Tu J. F., Wang L. Q. (2020). Acupuncture of different treatment frequencies in knee osteoarthritis: a pilot randomised controlled trial. *Pain*.

